# Perinatal mortality and its determinants in Sub Saharan African countries: systematic review and meta-analysis

**DOI:** 10.1186/s40748-020-00120-4

**Published:** 2021-01-01

**Authors:** Dawit Tiruneh, Nega Assefa, Bezatu Mengiste

**Affiliations:** 1 Department of Midwifery, College of Health Sciences, Debre Tabor University, National State of Amhara, Debre Tabor Town, South Gondar Province Ethiopia; 2 Department of Nursing, College of Health and Medical Science, Haramaya University, Harar, Ethiopia; 3 Department of Environmental Science, College of Health and Medical Science, Haramaya University, Harar, Ethiopia

**Keywords:** Perinatal mortality, Determinants, Random effect, Effect size, Heterogeneity, Publication Bias, Sensitivity, Sub-Saharan

## Abstract

**Background:**

Despite decreasing overall perinatal and maternal mortality in high-income countries, perinatal and maternal health inequalities are persisting in Sub Saharan African countries. Therefore, this study aimed to determine the effects size of rates and determinants for perinatal mortality in Sub-Saharan countries.

**Method:**

The sources for electronic datasets were PubMed, Medline, EMBASE, SCOPUS, Google, Google Scholar, and WHO data Library. Observational studies published in the English language from January 01, 2000, to May 30, 2019 were included. STROBE and JBI tools were used to include relevant articles for this review. We used a Comberehensive Meta-Analysis version 2 software for this analysis. The I^2^ and Q- statistic values were used to detect the level of heterogeneity. The Kendall’s without continuity correction, Begg and Mazumdar rank correlation and Egger’s linear regression tests were used to detect the existence of significant publication bias (*P* <  0.10). The effects size were expressed in the form of point estimate and odds ratio with 95% CI (*P* <  0.05) in the random effect analysis using the trim and fill method.

**Result:**

Twenty-one articles were included in this review. However, only fourteen studies reported the perinatal mortality rate. Among 14 studies, the observed and adjusted PMR was found to be 58.35 and 42.95 respectively. The odds of perinatal mortality among mothers who had no ANC visits was 2.04 (CI: 1.67, 2.49, *P* <  0.0001) as compared to those who had at least one ANC visit. The odds of perinatal mortality among preterm babies was 4.42 (CI: 2.83, 6.88, *P* <  0.0001). In most cases, heterogeneity was not evident when subgroup analyses were assessed by region, study design, and setting. Only perinatal mortality (P <  0.0001), antenatal care (*P* <  0.046) and preterm births (*P* <  0.034) showed a relationship between the standardized effect sizes and standard errors of these effects.

**Conclusion:**

In general, engaging in systematic review and meta-analysis would potentially improve under-represented strategies and actions by informing policy makers and program implementers for minimizing the existing socioeconomic inequalities between regions and nations.

## Background

Perinatal mortality is the best indicator of the quality of prenatal, delivery, and early infant care practices available in any circumstances. It contributed to 40% of deaths to overall under-five mortality [1, 2]. Reducing inequities and reaching the most vulnerable children are the emphases of all concerned bodies for ending preventable deaths of newborns and children under five years of age by 2030. According to the United Nations (UNs) reports in 2017, 1 in 36 infants die in the first month of life in sub-Saharan Africa as compared with 1 in 333 in high-income countries [2].

Maintaining an effective balance between preserving normality and ensuring a state of readiness in an attempt to reduce this gap represents a fundamental challenge to health systems and a tension in safe motherhood programming in Sub-Saharan countries [3–6]. Perinatal and maternal health inequalities are persistently high and remain beyond the acceptable level in low-income countries of Africa. In addition, perinatal mortality indicates the extent of pregnancy wastage and the quality and quantity of health care services available to the mother and the newborn [5]. Globally, an estimated 2.6 million stillbirths occur each year. Of these, half of them occur during labor and birth. Most stillbirths result from preventable conditions such as maternal infections, non-communicable diseases, and obstetric complications [6].

Ending preventable perinatal death is high on the international public health concern even though there is slow progress in preventing perinatal deaths [7]. However, improving people’s health and quality of life requires collective actions for equity of fair distribution of resources and addressing disparities of health inequities between regions, especially in rural and urban areas [8]. As part of the Early Neonatal Action Plan (ENAP), the World Health Organization (WHO) is developing a perinatal audit as a means to assist in addressing modifiable factors. Its focus is creating a link to a minimum perinatal dataset [9] after the UN 2030 agenda embraces good health is a precondition for outcome and measure of sustainable development program. The UN 2030 agenda is targeting to reduce MMR to less than 70 per 100,000 live births, NMR to less than 12/1000 live births, and under-five mortality rate to less than 25 per 1000 live birth [10]. In general, collective efforts and actions taken into account in the era of sustainable development programs should be implemented based on the nation’s cultural, economic, and societal contexts.

Although there are discrepancies between studies in Sub-Saharan regions, no systematic review or meta-analysis studies exist in the study area. This review allows health care providers, researchers, and policymakers to efficiently integrate existing information and provide data for decision-making in the most relevant context of perinatal health. Therefore, the current systematic review and meta-analysis aimed to determine the pooled estimate of the perinatal mortality rate and the effects sizes of determinants for perinatal mortality. It aims to help identify the root causes of discrepancies between studies in Sub Saharan African countries.

## Method

### Search strategy

Studies for this review and meta-analysis were accessed in electronic web-based searches using different search engines. Published articles in the English language were intensively accessed and examined to minimize the level of publication and selection bias. The sources for electronic datasets were PubMed, Medline, EMBASE, SCOPUS, Google, Google Scholar, and WHO data Library. The ancestor search strategy was accessed, aiming to arrive at the final number of studies. Studies that were cited by others were also looked online (descendent search strategy). In combination with MeSH terms, we used the Boolean operator ‘AND’ and ‘OR’ to connect and focus a search from Pubmed. The search terms we used include *‘incidence, prevalence, rate, ratio, risk factors, determinant, perinatal mortality, perinatal death, stillbirth, early neonatal death and sub-Saharan’* (Table 1).

**Table 1:** Pubmed search strategies and search details for perinatal mortality and its determinants

S. No.	Search terms and strategies	Examples of search details
**1**	Incidence/prevalence AND rate/ratio	*“(((Incidence/prevalence[All Fields]AND(“risk factors “[MeSH Terms] OR (“risk”[All Fields] AND “factors”[All Fields]) OR “risk factors”[All Fields] AND determinant[All Fields] AND (“perinatal mortality”[MeSH Terms] OR (“perinatal”[All Fields]*))*)”*
**2**	Risk factors AND/OR determinant	
**3**	Perinatal mortality AND/OR perinatal death	
**4**	Outcome/death AND/OR still birth	
**5**	Early neonatal death AND/OR neonatal death	
**6**	Sub AND Saharan	

### Eligibility criteria

The methodological qualities and the outcome of each study was critically examined in the review process. Studies were included in the review if the study:

- was conducted on perinatal mortality in non-Arab state members of the Sub-Saharan countries in Africa
- was published in the English language from January 01, 2000, to May 30, 2019 Gregorian calendar (GC)
- was observational study design
- design was cross-sectional, case-control or cohort
- was conducted based on the definition of classification for perinatal mortality and its determinants

### Definition of the outcome of interest

The outcomes of interest in this review were perinatal mortality and eight selected determinants of perinatal mortality in Sub-Saharan African countries.

- The perinatal period: It commences at 28 completed weeks (154 days) of gestation and ends seven completed days after birth.
- The perinatal mortality rate: The sum of stillbirth rate and early neonatal mortality rate within the first week of life
- *Stillbirth: A baby born with no signs of life at or after 28 weeks’ gestation* or birth weight of 1000 g or more or body length of 35 cm or more [1]

### Study identification and selection

During the data extraction process, we used the reviewers’ manual data extraction form that has been developed by the 2014 JBI institute. The information on the title, author, publication year, study design, sample size, study participants, sampling methods, and outcome of interest were considered in the selection process. The first author conducted the primary searching of studies from different sources. Initially, our colleagues (AA and SB) searched and identified potential articles using predetermined selection criteria. Following the identification, DT made the final selection through a critical review of full-text articles. Co-authors (NA and BM) closely supervised the selection process. In this review, we excluded full-text articles that failed to report sufficient sample statistics or raw data. In general, no study was excluded without a thorough evaluation using STROBE critical appraisal [11] and JBI quality assessment tools [12]. The final quality score was set for each study design by discussion.

### Data abstraction

This review was conducted from June 01, 2019, to July 24, 2019, using the STROBE critical appraisal tools. We further assessed studies using the checking points in the JBI quality assessment tool. For each study design, we included a study that scored above the mean value of the checking points. We used the preferred reporting Item for Systematic Review and Meta-Analyses (PRISMA 2009) to arrive at the final 21 included articles [13].

We assessed the study objectives, designs, period, location, settings, generalizability, and relevance to the study population of the primary articles. Statistically significant variables and statistical analysis models on topics related to the current research were extracted, retrieved, and included. After removing duplicated studies, we excluded irrelevant articles’ titles and abstracts. Then, we excluded abstracts that failed to show relationships of associated variables with perinatal mortality. Finally, we excluded full-text studies which did not fulfill the predetermined criteria of the review.

### Heterogeneity

We assessed the presence of heterogeneity using the Chi-square statistic (Cochran’s-Q), Tau (τ^2^) and I-squared (I^2^) with their corresponding *P*-value. We used the Chi-square statistic (Q) to determine the extent of heterogeneity across studies. A Q – statistic more than the chi-square value corresponding to the degree of freedom, and *P* <  0.05 indicates the presence of heterogeneity [14, 15]. The τ^2^ and I^2^ statistics were used to assess the heterogeneity of studies within and between studies, respectively [16]. We determined the extent of heterogeneity as mild (25%), moderate (50%), and high (75%) heterogeneity. An I^2^ of zero means that all variability in effects size estimates is due to sampling error within studies [17, 18].

### Publication bias

We assessed the presence of publication bias using the funnel plot asymmetry, the Begg and Mazumdar rank correlation and Egger’s linear regression. Using the visual presentation of the funnel plot for detecting asymmetry and the Kendall’s S statistics score (P-Q) for showing the direction of the correlation were subjective to detect the presence of publication bias. Therefore, the *τ*^*2*^ statistical significance (*P* <  0.10), Kendall’s without continuity correction and Egger’s linear regression tests were used to detect the possible existence of significant publication bias (*p* <  0.10) at a 95% confidence interval for statistical analysis [16, 19–21].

### Sensitivity analysis

In this study, the robustness of the findings were examined through sensitivity analysis. It was used to assess the presence of publication bias, the effect of study quality, and the results of the effect size. We conducted a sensitivity analysis with large and small effect size outliers using inferential statistics of this meta-analysis [22, 23]. Regarding removing one sample, we repeated the meta-analysis multiple times, each time leaving out one sample to analyze the distribution mean change when a given sample is excluded from the analysis considering the results of influential samples [24].

### Statistical analysis

We used an excel sheet to extract and organize the necessary information from each original study. Both the observed and adjusted point estimates were expressed in the form of event rate per 1000 total births for perinatal mortality and odds raios with the associated 95% CI in the random-effects model. The random-effects model was selected to estimate the pooled effect size of the perinatal mortality rate and its purposely selected determinants using a Comprehensive Meta-Analysis (CMA) version 2 software [25]. The model assumes that primary studies might differ in the implementations of interventions and selection of participants. Also, the effect sizes in the original studies might represent a random sample from a particular distribution of these effects size [16].

Also, to test the statistical significance of differences between groups and compare the mean effects of two or more groups, subgroup analyses were conducted using regions, study settings, and designs [26]. The adjusted effect size was determined by applying Duval and Tweedie’s trim and fill method in the random-effects analysis [27]. Duval and Tweedie’s procedure stated that if the point estimate was to be adjusted for bias left or right of the mean, it would remain unchanged for the random-effects model [16]. Forest plot, high resolution, and funnel plot tests displayed the results of the mean effect sizes in the form of event rate and odds ratio.

## Result

### Systematic review results

A total of 351 articles were retrieved through electronic searching by titles and abstracts. Of these records, we arrived at 21 eligible studies to estimate the observed and adjusted effect sizes, the extent of heterogeneity, and the existence of publication bias for perinatal mortality rate and its selected determinants (Fig. 1).

**Fig. 1:** Steps of selecting relevant articles using the PRISMA Group (Moher et al., 2009). Preferred Reporting Items for Systematic Reviews and Meta-Analyses

### Description of studies

Of the 21 included studies, eight were cross-sectional, six were case-control, and seven were cohort studies. Regarding the study setting, eleven were in the facility, eight were in the community, and only two were population-based studies. These review included studies from Ethiopia [28–32], Nigeria [33–36], Tanzania [37, 38], Zimbabwe [5, 39], Uganda, Ghana [40], Côte d’Ivoire [41], Burkina Faso [42], Kenya [43], Rwanda [44], Malawi [45], and Mozambique [46]. Most studies in Ethiopia and Nigeria were eligible and presented in this review. We included studies published from 2000 to 2019 Gregorian Calendar (GC), and the sample size ranges from 378 in Ethiopia [31] to a maximum of 25,817 in Nigeria [33]. Ethiopia [30] and Uganda reported the lowest and the highest perinatal mortality rate, respectively. Overall, studies included in this review have a total sample size of 118,372 pregnant mothers in the Sub-Saharan region (Table 2).

**Table 2:** Characteristics of included articles for systematic review for perinatal mortality rate in Sub-Saharan countries, 2000–2019 Gregorian Calendar (GC)

Author, Year	R	S	D	SS	Determinants	Association with PMR AOR(95% CI)	PMR
Getiye et al., 2017, [28] Ethiopia	EA	FB	CC	1113	Short birth interval	4.55 (1.79–11.54)	NR
					Preterm Delivery	2.02 (1.08–3.77)	
					Hx of perinatal loss	6.36 (1.51–26.76)	
					Low Birth weight	16.45 (9.57–28.26)	
Aragaw YA, 2016, [29] Ethiopia	EA	FB	CS	3786	No ANC visit	2.05 (1.48–2.87)	98.2
					Shoulder delivery	5.95 (2.11–16.86)	
					Breech delivery	4.06 (1.856–8.912)	
					Low birth weight	5.03 (1.63–15.00)	
Yirgu R et al., 2016, [30] Ethiopia	EA	CB	CC	4097	Primipara	3.15 (1.03–9.60)	25.1
					Hx of perinatal loss	2.46 (1.03,5.86)	
					Hx of perinatal loss	9.55 (4.67–19.54)	
					Preterm birth	9.44 (1.81–49.22)	
Goba et al. 2018, [31] Ethiopia	EA	FB	CC	378	Preterm birth	12.2 (3.46, 43.17)	NR
	Z				Low birth weight	11.5 (3.16–42.36)	
					No ANC visit	5.4 (0.80–36.63)	
					Short birth interval	2.2 (1.03–5.09)	
Andargie et al. 2013, [32] Ethiopia	EA	CB	Co	1752	Hx of perinatal loss	8.38 (3.94, 17.83)	50.22
					Multiple gestation	7.09 (3.22, 15.61)	
					Short birth interval	2.58 (1.61, 4.13)	
Nkwo et al., 2014, [33] Nigeria	WA	PB	CS	25,817	Hx of perinatal loss	3.31 (2.73, 4.02	36
					Multiple gestation	3.12 (2.11, 4.59)	
					Short birth interval	1.65 (1.26, 2.17)	
					Low birth weight	2.57 (1.79, 3.69)	
Fawole et al., 2011, [34] Nigeria	WA	FB	CS	9177	No ANC visit	1.74 (1.27, 2.39)	78
					Preterm birth	1.89 (1.12, 3.19)	
					Elective CS	0.12 (0.05, 0.36)	
					Emergency CS	0.73 (0.55, 0.96)	
Owolabi et al. 2008,	WA	FB	Co	894	Primipara	0.67 (0.26, 1.73)	NR
[35] Nigeria							
Ekure et al. 2011, [36] Nigeria	WA	FB	CS	560	Primipara	^c^ 0.07 B (0.02, 0.06)	84.6
					Low birth weight	^c^ − 0.09 B(− 0.05, 0.02)	
Schmiegelow et al. 2012, [37] Tanzania	EA	CB	Co	872	Preterm birth	14.47 (3.23, 64.86)	NR
Habib et al. 2008, [38] Tanzania	EA	FB	CS	15,255	Preterm birth	^a^ 2.2 (1.7, 2.8)	43.9
Feresu et al. 2005, [39] Zimbabwe	SA	FB	CS	15,117	No ANC visit	^b^ 2.52 (1.63, 3.91)	65
					Primipara	^b^ 1.52 (0.97, 2.38)	
					Breech Delivery	^b^ 10.53 (6.78, 6.34)	
					Instrument delivery	^b^ 3.38 (1.64, 6.96)	
Tachiweyika et al. 2011, [5] Zimbabwe	SA	CB	CC	10,540	Low birth weight	9.46 (3.91, 27.65)	NR
Moyer et al. 2016, [40] Uganda	WA	CB	CS	4883	–	–	105.88
Engmann et al. 2012, [41] Ghana	WA	PB	CS	17,300	Primipara	1.75 (1.28, 2.40)	39
					Preterm birth	2.84 (2.11, 3.81)	
					Multiple gestation	5.22 (3.61, 7.54)	
Kone et al., 2018, [42] *Côte d’Ivoire*	WA	CB	Co	2976	Hx of perinatal loss	23.2 (14.71, 36.55)	33
					Preterm birth	4.45 (2.82, 7.01)	
					Caesarean section	13.03 (4.24, 40.08)	
					Instrument delivery	5.05 (1.50, 16.96)	
Diallo et al. 2010, [43] Burkina Faso	WA	CB	Co	895	Primipara	2.20 (1.2, 3.9)	79
					Multiple gestation	^b^ 4.0 (2.3, 6.9)	
Yego et al. 2014, [44] Kenya	EA	FB	CC	600	No ANC visit	4.5 (1.2, 16.7)	NR
					Preterm birth	7.0 (2.4, 20.4)	
					Low birth weight	6.6 (3.8, 10.2)	
Musafili et al. 2015, [45] Rwanda	EA	FB	CC	672	–	–	32
kulmala et al. 2000, [46] Malawi	EA	CB	Co	780	Cesarean section	^b^ 4.4 (1.4, 13.9)	NR
					Hx of perinatal loss	^b^ 2.7 (1.3, 5.7)	
N.B Osman et al. 2001, [47]	SA	FB	Co	908	Preterm birth	8.48 (3.44, 20.90)	47
Mozambique					Low Birth weight	AOR 4.20 (1.49–11.86)	

Association with PMR reported as adjusted odds ratio (95% confidence interval) except as noted ^a^ relative risk, ^b^Adjusted Relative risk, and ^c^Standard coeffiecent,

Region (R) is coded: *EA* East Africa, *SA* South Africa, *WA* West Africa., Study type is coded, *CB* Community Based, *FB* Facility Based, *PB* Population Based, Study design is coded, *CC* Case control, *Co* Cohort, *CS* Cross Sectional, Sample size (SS) is coded, Perinatl mortality rate (PMR) is coded, *NR* Not Reported

### Perinatal mortality

Of the 21 eligible studies, only fourteen studies reported perinatal mortality rates in the Sub-Saharan region and the reports showed us discrepancies of perinatal mortality rate in Sub-Saharan countries. All fourteen studies reporting perinatal mortality rate were eligible and included in the meta-analysis to assess the pooled effects size of the perinatal mortality rates. The overall observed perinatal mortality rate was 58.35 (95% CI: 46.19, 70.51, *P* <  0.0001) per 1000 total births (stillbirth and live births) in the random-effect analysis (Fig. 2). Four studies were slimmed to estimate the adjusted effect sizes of perinatal mortality rates in Sub-Saharan countries (Pooled PMR: 42.95, 95% CI: 29.21, 56.70).

**Fig. 2:** Forest plot of perinatal mortality rate in Sub-Saharan countries, 2000–2019 GC

### Subgroup analysis and perinatal mortality

We conducted subgroup analyses to estimate the mean effect sizes of perinatal mortality in three regions of Africa (West Africa, East Africa, and South Africa). Studies in West Africa showed the highest perinatal mortality rate, 65.07 (95% CI: 47.07, 83.07) as compared to studies in East Africa, 49.88 (95% CI: 28.59, 71.18), and South Africa, 56 (95% CI: 22.33, 89.67). The rates were high in a facility-based study setting, 64.09 (95% CI: 46.00, 82.2), and cross-sectional study design, 68.82 (95% CI: 53.83, 83.81). The I^2^ test showed high levels of heterogeneity by region, study setting, and study design with a strong statistical significance (*P* <  0.001) (Table 3).

**Table 3:** Subgroup analysis of perinatal mortality rate by region, study setting and design in Sub-Saharan countries, 2000–2019 GC

Sub group	Number of studies	PMR (95% CI)	Standard error	P-value (P)	Extent of heterogeneity		
					I^2^	Q- stat	P-value (P)
Region							
E. Africa	5	49.88 (28.60, 71.18)	10.86	< 0.0001	99.99	47,751	< 0.0001
S. Africa	2	56.00 (22.33, 89.67)	17.18	< 0.001	99.96	2893	< 0.0001
W. Africa	7	65.07 (47.07, 83.07)	9.18	< 0.0001	99.99	79,902	< 0.0001
Setting							
CB	5	58.64 (37.22, 80.06)	10.93	< 0.0001	99.99	70,302	< 0.0001
FB	7	64.09 (46.00, 82.20)	9.24	< 0.0001	99.99	58,306	< 0.0001
PB	2	37.50 (3.63, 71.36)	17.28	< 0.03	99.17	120	< 0.0001
Design							
CS	8	68.82 (53.83, 83.81)	7.65	< 0.0001	99.99	79,476	< 0.0001
CC	2	28.55 (−1.43, 58.53)	15.30	> 0.062	99.88	834	< 0.0001
Co	4	52.30 (31.10, 73.50)	10.82	< 0.0001	99.98	19,084	< 0.0001

### Sensitivity analysis and perinatal mortality

We conducted a sensitivity analysis to reduce the level of heterogeneity between studies. We removed some outlier studies having small and high relative weight. Because they might potentially affect the estimation of the true effect size. Two studies in Ethiopia [30] and Uganda [39] showed the highest (13.69%) and the smallest relative weight (3.24%) respectively. When these studies were excluded and running the analysis, the cumulative perinatal mortality rate was slightly lowered to 57.16 (45.67, 68.65, *P* <  0.0001). Similarly, when we performed removing one study in the meta-analysis using the CMA software, the CI of each became narrower. However, we did not see a change in the overall rate of perinatal mortality (Fig. 3).

**Fig. 3:** Forest plot of sensitivity analysis when one study of perinatal mortality revomed from Meta-Analysis in Sub-Saharan countries, 2000–2019 GC

### Determinants and perinatal mortality rate

In the random-effects analysis, we purposely selected only eight determinants from 21 eligible studies of perinatal mortality in Sub-Saharan countries. These were low birth weight less than 2500 g, primiparity, presence of ANC visits, history of abortion or perinatal loss, multiple gestation (two or more), preterm birth less than 37 completed weeks, birth interval less than two years, and mode (non-spontaneous) of delivery. There was a statistically significant association between these determinants and perinatal mortality in the study region.

### Low birth weight and perinatal mortality

In this meta-analysis, seven studies [5, 28–30, 36, 43, 46] were included. The observed odds ratio of low birth weight for the risk of perinatal mortality was 8.69 (CI: 6.04, 12.51, *P* <  0.001) as compared to babies born with an adequate birth weight (2500-3999 g) (Table 4). In this analysis, observed and adjusted effect sizes of low birth weight were equal, revealed no studies were slimmed to adjust publication bias. However, there was a moderate level of heterogeneity in the study region (I^2^: 35.19, Q: 9.26, *P* >  0.16). In the subgroup analysis by region, there was a moderate level of heterogeneity in East African studies (I^2^: 56.72, Q: 6.93, *P* >  0.74). However, it was not evident in total studies by region (Q: 0.44, df: 2, *P* > 0.802), study setting (Q: 0.032, df: 2, *P* > 0.859) and study design (Q: 2.166, df: 2, *P* > 0.339).

**Table 4:** High resolution plot of the odds of low birth weight for perinatal mortality rate in Sub-Saharan Countries, 2000–2019 GC

NB: Favors ‘A’: Normal birth weight, Favors ‘B’: Low birth weight

### Primiparity and perinatal mortality

In this category of meta-analysis, five studies [35, 36, 39, 40, 42] were included. The observed odds ratio of primiparity for the risk of perinatal mortality was 1.56 (CI: 1.18, 2.05, *P* <  0.002) (Table 5). As for birth weight, observed and adjusted values were equal revealing that no studies were slimmed to estimate the final effect sizes of primiparity for perinatal mortality. A moderate level of heterogeneity was observed (I^2^: 32.06, Q: 5.89, df: 4, *P* > 0.208). In subgroup analysis, a moderate level of heterogeneity was observed in West African studies (I^2^: 45.15, Q: 5.47 df: 3, *P* > 0.14), facility-based studies (I^2^: 56.66, Q: 4.62, df: 2, P > 0.1) and cohort study designs (I^2^: 71.43, Q: 3.50, df: 1, *P* > 0.061). But, it was not evident in total studies by region (Q: 0.395, df: 1, *P* > 0.53), study setting (Q: 0.95, df: 2, *P* > 0.623) and study design (Q: 0.19, df: 1, *P* > 0.664).

**Table 5:** High resolution plot for the odds of primiparity for perinatal mortality rate in Sub-Saharan Countries, 2000–2019 GC

NB: Favors ‘A’: Multipara, Favors ‘B’: Primipara

### ANC visits and perinatal mortality

Five studies [29, 31, 34, 39, 43] were included in this meta-analysis. The observed odds ratio of no ANC visit was 2.04 (CI: 1.67, 2.49, *P* <  0.001) for the risk of perinatal mortality as compared to those who had at least one ANC v**isit** (Table 6). Two studies were filled to estimate the adjusted effect sizes of ANC visits (POR: 1.99, CI: 1.60, 2.46). In this category of meta-analysis, we only detected a mild level of heterogeneity in East Africa studies (I^2^: 7.27, Q: 2.16, df: 2, *P* > 0.34).

**Table 6:** High resolution plot of the odds with No ANC visits for perinatal mortality rate in Sub-Saharan Countries, 2000–2019 GC

NB: Favors ‘A’: At least one ANC visit, Favors ‘B’: with No ANC visits

### History of perinatal loss and perinatal mortality

Five studies [28, 30, 32, 33, 41] were included. The observed odds ratio of history of perinatal loss for the risk of perinatal mortality was 8.34 (CI: 3.15, 22.1, *P* <  0.001) as compared to those mothers who had no history of perinatal loss (Table 7). Three studies were trimmed to estimate the adjusted effect size of the history of abortion or perinatal loss (POR: 3.57, CI: 1.44, 8.81). In this case, a high level of heterogeneity was observed (I^2^: 98.32, Q: 59.54, df: 1, P <  0.001). In subgroup analysis, a high level of heterogeneity in West African studies (I^2^: 98.32, Q: 59.54, df: 1, *P* <  0.001). Both community (I^2^: 72.67, Q: 7.317, df: 2, *P* <  0.026) and cohort studies (I^2^: 80.48, Q: 5.12, df: 1, *P* <  0.024) showed a moderate level of heterogeneity. However, its heterogeneity was not evident in total studies by region (Q: 0.003, df: 1, *P* > 0.957). It reduced to mild level by setting (Q: 4.58, df: 2, *P* > 0.101) and design (Q: 5.03, df: 2, *P* > 0.081).

**Table 7:** High resolution plot of the odds of history (Hx) of perinatal loss for perinatal mortality rate in Sub-Saharan Countries, 2000–2019 GC

NB: Favors ‘A’: no history (Hx) of perinatal loss, Favors ‘B’: With history (Hx) of perinatal loss

### Multiple gestation and perinatal mortality

Five studies [32, 33, 38, 40, 42] were included for this meta-analysis. The observed odds ratio of multiple gestations (twin and more) for the risk of perinatal mortality was 3.85 (CI: 2.60, 5.71, *P* <  0.001) as compared to mothers with a singleton pregnancy (Table 8). Two studies were slimmed to estimate the adjusted effect size of multiple gestation for perinatal mortality (POR: 2.97, CI: 1.20, 4.43). There was a high level of heterogeneity in the region (I^2^: 77.25, Q: 17.58, df: 4, *p* <  0.001). This determinant was highly heterogeneous in East Africa studies (I^2^: 85.51, Q: 6.90, df: 1, *P* <  0.009). There were high (I^2^: 91.90, Q: 12.35, df: 1, P <  0.001) and moderate (I^2^: 48.34, Q: 1.94, df: *P* > 0.16) level of heterogeneity in facility and community based studies respectively. Similarly, there were high (I^2^: 85.84, Q: 14.12, df: 2, P <  0.001) and moderate (I^2^: 48.34, Q: 1.94, df: 1, P > 0.16) level of heterogeneity in cross section and cohort studies respectively. However, heterogeneity was not evident in total studies by region (Q: 0.39, df: 2, *P* > 0.822), setting (Q: 0.28, df: 2, *P* > 0.870) and design (Q: 0.39, df: 1, *P* > 0.532).

**Table 8:** High resolution plot of the odds of multiple gestation as a determinant for perinatal mortality rate in Sub-Saharan Countries, 2000–2019 GC

NB: Favors ‘A’: No nultiple gestation, ‘B’: multiple gestation

### Preterm birth and perinatal mortality

Nine primary studies [28, 30, 31, 34, 37, 40, 41, 43, 46] were included. The observed odds ratio of preterm babies whose gestational age was less than 37 completed weeks was 4.42 (CI: 2.83, 6.88, *p* <  0.001) for the risk of perinatal mortality as compared to term babies (Table 9).

**Table 9:** High resolution plot of the odds of preterm birth as a determinant for perinatal mortality rate in Sub-Saharan Countries, 2000–2019 GC

NB: Favors ‘A’: Term birth (37–42 weeks of gestation), Favors ‘B’: Preterm birth (less than 37 completed weeks)

Two studies were trimmed to estimate the adjusted effect size of preterm birth on perinatal mortality (POR: 3.31, CI: 2.10, 5.22). There was a moderate level of heterogeneity (I^2^: 69.43, Q: 26.172 df: 8, *P* <  0.001). In sub group analysis, a moderate level of heterogeneity in East Africa was observed (I^2^: 71.08, Q: 13.83 df: 4, *P* <  0.008). There was a moderate level of heterogeneity in facility studies (I^2^: 77.72, Q: 17.95, df: 4, P <  0.001) and cross-sectional study design (I^2^: 72.76, Q: 11.013, df: 3, *P* <  0.012). However, heterogeneity was not evident in total studies by region (Q: 3.69, df: 2, *P* > 0.158), setting (Q: 1.08, df: 2, *P* > 0.582) and design (Q: 4.13, df: 2, *P* > 0.127).

### Birth interval and perinatal mortality

Four primary studies [28, 31–33] were included. The observed odds ratio of birth interval was 2.24 (CI: 1.53, 3.29, *P* < 0.0001) for the risk of perinatal mortality as compared to babies born where birth interval was two or more years (Table 10). Two studies were trimmed to estimate the adjusted effect size of short birth interval (< 2 years) for the risk of perinatal mortality (POR: 1.75, CI: 1.18, 2.60). There were moderate level of heterogeneity (I^2^: 50.62, Q: 6.07 df: 3, *P* > 0.108). In sub group analysis, heterogeneity was not evident in East Africa (I^2^: 0, Q: 1.52, df: 2, *P* > 0.468). Both facility setting studies and case control study designs showed a mild and equal level of heterogeneity (I^2^: 28.80, Q: 1.4, df: 1, *P* > 0.236). But, there was no evidence of heterogeneity between total studies by region (Q: 4.56, df: 2, *P* < 0.033) or by study setting and design with equal statistical values (Q: 1.79, df: 2, *P* > 0.408).

**Table 10:** High resolution plot of the odds of short birth interval as a determinant for perinatal mortality rate in Sub-Saharan Countries, 2000–2019 GC

NB: Favors ‘A’: Normal birth interval, Favors ‘B’: Short birth interval (less than two years)

### Mode of deliveries and perinatal mortality

Among four included studies [30, 34, 39, 41], there were seven statistical associations from five determinants; two instrumental, one emergence Cesarean Section, one elective Cesarean Section, two breech, and one shoulder delivery. One included study has more than one statistical association making a total of seven independent odds ratio. The odds ratio of these determinants among mothers who gave birth through non-spontaneous vaginal delivery was 2.94 (CI: 0.99, 8.72, *P* > 0.052) as compared to mothers who gave birth through spontaneous vaginal delivery (Table 11). Three studies were trimmed to estimate the adjusted effect size of non-spontaneous mode of delivery for perinatal mortality (POR: 1.20, CI: 0.39, 3.68). There was a high level of heterogeneity (I^2^: 95.40, Q: 152.22, df: 7, *P* < 0.0001). In sub group analysis by region, there was a moderate level of heterogeneity (I^2^: 50.62, Q: 6.07 df: 3, *P* > 0.108). There was a high level of heterogeneity in West Africa (I^2^: 93.23, Q: 44.32, df: 3, P < 0.0001), in facility studies (I^2^: 96.36, Q: 137.56, df: 5, P < 0.0001) and cross-sectional study designs (I^2^: 96.36, Q: 137.56, df: 5, P < 0.0001). But, it was not evident in total studies by region (Q: 1.89, df: 3, *P* > 0.595), study setting and design (Q: 1.053, df: 1, *P* > 0.305).

**Table 11:** High resolution plot of the odds of non-spontaneous vaginal delivery for perinatal mortality rate in Sub-Saharan Countries, 2000–2019 GC

NB: Favors ‘A’: Spontaneous vaginal delivery, Favors ‘B’: Non-spontanous delivery (Instrumental, Cesarean, Emergence Cesarean, Elective Cesarean, Shoulder, and breech delivery).

## Discussion

In this systematic review and meta-analysis, the overall observed perinatal mortality rate was 58.35 (95% CI: 46. 19, 70.51, *P* < 0.001) per 1000 total births in the random-effect analysis. Four fitted values made the adjusted effect size of PMRs to be 42.95 (95% CI: 29.21, 56.70). We also conducted subgroup analyses to compare the difference between effect sizes in different groups. In this subgroup of meta-analysis, the PMRs were high in West Africa, 65.07 (95% CI: 47.07, 83.07), in a facility setting, 64.09 (95% CI: 46.00, 82.20) and as reported in studies using cross-sectional study design, 68.82 (95% CI: 53.83, 83.81).

### Heterogeneity and publication bias in perinatal mortality

There was heterogeneity of studies in reported PMRs and their determinants. Its extent was high in the study region (I^2^: 99.99, df: 13, Q: 143573.67, *P* < 0.0001). Both the I-squared (I^2^) and Cochran (Q) tests showed high levels of heterogeneity in each study by region, study setting, and study design with a strong statistical association (*P* < 0.001). However, it was not evident in total studies by region (Q: 1.16, df: 2, *P* > 0.56), setting (Q: 1.84, df: 2, *P* > 0.398) and design (Q: 5.982, df: 2, *P* > 0.05) using subgroup analyses. The possible reason for this bias could be the inclination of researchers in reporting findings only achieving statistical significance. It might lead to inaccurate conclusions in a meta-analysis that could seriously impact the clinical practices.

Begg and Mazumdar’s test estimated the rank correlation (Kendall’s) between the standardized Effect Sizes (ES) of PMRs and variances or standard errors (SE) of these effects. It may be interpreted much the same way as any correlation, with a value of zero indicating no relationship between effect size and precision. If the value (P-Q) deviates from zero, it subjectively informs us the presence of a relationship. An asymmetry of funnel plot exists when large standard errors are associated with larger effect sizes. The possible causes of this relationship may be the presence of publication bias [16, 19–22, 47]. The size of the intercept provides a measure of asymmetry - the larger the deviation from zero, the greater the asymmetry. A positive intercept indicates that the effect estimated from the smaller studies is greater than the effect estimated from larger studies. Conversely, a negative intercept indicates that the effect estimated from the smaller studies is less than the effect estimated from larger studies [16, 19, 22].

In this meta-analysis of the PMRs, Begg and Mazumdar rank correlation revealed a Kendall’s S statistic was deviated from zero (P-Q = 91), and Kendall’s Tau (τ) without continuity correction = 1.00 (*P* < 0.0001). In addition, the Egger’s linear regression intercept (469.94, 95% CI: 441.63, 498.25, P < 0.0001) did not include zero indicating the presence of a relationship. It implies that there was evidence of heterogeneity and publication bias in Sub-Saharan studies of perinatal mortality. However, it was not evident in subgroup analysis using region, setting, and study design. In this meta-analysis, missed studies were fitted on the left side of the mean value of the effect sizes during analysis athough it has no effect in the random effect model. However, smaller effects size in the left direction is more likely favored in the publication process and studies with large effects size may be suppressed to the right from the median line of the funnel plot [16, 19, 27].

In this study, both Begg’s rank correlation and Egger’s regression tests confirmed the presence of a relationship between the standardized effect sizes and the standard error of these effects. Publication bias might be the cause of the relationship. In this analysis of PMRs, the visual presentation of the funnel plot was asymmetric and skewed in a positive direction. However, four studies were fitted in a negative direction to treat the asymmetry. This asymmetry might occur due to the existence of publication bias (Fig. 4).

**Fig. 4:** Funnel plot of standard error by perinatal mortality rate in Sub-Saharan countries, 2000-2019 GC

### Determinants for perinatal mortality

In this subcategory of meta-analysis, observed and adjusted values of low birth weight for the risk of perinatal mortality were equal and revealed that publication bias did not exist. Begg and Mazumdar rank correlation revealed a Kendall’s S statistic was closed to zero (P-Q = − 1), and Kendall’s Tau (τ) without continuity correction = − 0.048 (*P* > 0.881). The Egger’s regression test did also include zero (Intercept: -1.48, 95% CI: − 5.373, 2.421, *P* > 0.375). Therefore, both methods revealed no relationship between the standardized ESs and SE of these effects. Similarly, the adjusted values for primiparity was equal to the observed values to estimate the final effect sizes. Begg and Mazumdar rank correlation revealed a Kendall’s Significance (S) statistic was deviated from zero (P-Q = − 10), and Kendall’s Tau (τ) without continuity correction = − 1.00 (*P* < 0.014). However, the Egger’s regression test revealed no relationship between the standardized ESs and SE of these effect sizes because the intercept did include zero (Intercept: -2.42, 95% CI: - 6.01, 1.16, *P* > 0.12).

Regarding the ANC visits, two studies were slimmed to estimate the effect sizes of no ANC visits for the risk of perinatal mortality. Begg and Mazumdar rank correlation revealed a Kendall’s S statistic was deviated from zero (P-Q = 8), and Kendall’s Tau (τ) without continuity correction = 0.80 (*P* < 0.05). The Egger’s regression did not include zero (Intercept: 1.57, 95% CI: 0.05, 3.08, *p* < 0.046). Therefore, both methods showed us the presence of relationships between the standardized ESs and SE of these effect sizes. Three studies were trimmed to estimate the effect size of abortion or perinatal loss as a risk factor for perinatal mortality. Begg and Mazumdar rank correlation revealed a Kendall’s S statistic was closed to zero (P-Q = − 2), and Kendall’s Tau (τ) without continuity correction = − 0.20 (*P* > 0.624). The Egger’s regression did include zero (Intercept: 3.81, 95% CI: − 5.05, 12.68, *p* > 0.265). Both methods revealed no relationship existed.

Regarding multiple gestation, two studies were slimmed, and Begg and Mazumdar rank correlation revealed a Kendall’s S statistic was closed to zero (P-Q = 2), and Kendall’s Tau (τ) without continuity correction = 0.20 (P > 0.624). The Egger’s regression intercept did include zero (Intercept: 2.39, 95% CI: − 5.09, 9.88, *P* > 0.384). Therefore, both methods showed us the absence of a relationship. Likewise, three studies were trimmed to estimate the adjusted effect size of preterm birth on perinatal mortality. Begg and Mazumdar rank correlation revealed a Kendall’s S statistic was deviated from zero (P-Q = 8), and Kendall’s Tau (τ) without continuity correction = 0.22 (*P* > 0.404). The Egger’s regression intercept did not include zero (Intercept: 2.26, 95% CI: 0.22, 4.30, *P* < 0.034) and revealed the presence of a relationship. Publication bias might be the cause for this relationship.

Again, two studies were trimmed to estimate the size of the adjusted effect of birth interval less than two years for the risk factor of perinatal mortality. Begg and Mazumdar rank correlation revealed a Kendall’s S statistic (P-Q = 4) was closed to zero, and Kendall’s Tau (τ) without continuity correction = 0.67 (*P* > 0.174). The Egger’s regression did include zero (Intercept: 2.41, 95% CI: − 1.73, 6.55, *p* > 0.129). Therefore, both methods revealed no relationship. Finally, three studies were trimmed to estimate the size of the adjusted effects of non-spontaneous vaginal delivery for the risk of perinatal mortality. Begg and Mazumdar rank correlation revealed a Kendall’s S statistic was zero as expected (P-Q = 0), and Kendall’s Tau (τ) without continuity correction = 0.00 (*P* = 1.000). The Egger’s regression did include zero as expected (Intercept: 3.34, 95% CI: - 4.54, 11.22, *P* > 0.3397). Consequently, both methods showed that a relationship did not exist.

In general, studies would differ in design and conduct as well as in participants, interventions, exposures, or outcomes. It might be the possible reason in which most heterogeneity tests confirmed the presence of variation in effect sizes in this meta-analysis. It would also be the existence of the different studies caused by a systematic difference between the included studies for this review. Statistical heterogeneity exists when the effects differ between studies [47, 48]. A small number of included studies have a precision close to zero due to their large size effects. In this case, the funnel plot is supposed to be asymmetrical, and publication bias appears. For this purpose, we selected the trim-and-fill method to detect the significance of publication bias because we only reviewed twenty-one studies. It also provides bias-adjusted results for small studies [49–51] considering extracting unpublished studies is not achievable. This method estimates the size of the adjusted effects only by approximating statistically imputed missing values [27].

In this regression analysis, a positive intercept implies a bias towards the right side of the funnel plot, and the missing studies are in the negative direction. In contrast, a negative intercept indicates a bias toward the left side, and the missing values are likely in the right direction [22]. In this meta-analysis, the results obtained from small studies scattered widely at the bottom of the graph of the funnel plot. The spread was narrow at the top of the funnel plot of studies with adequate sample size [52]. In primiparity, the funnel plot was resembled a symmetrical graph showing the absence of publication bias**.** However, the results of most determinants for perinatal mortality were asymmetrically skewed to the positive direction indicating the presence of publication bias. The adjusted result of preterm birth was skewed in a positive direction, and some studies were slimmed to estimate the size of the adjusted effects. The possible reason might be missing studies suppressed by publication bias in a meta-analysis (Fig. 5).

**Fig. 5:** Funnel plot of standard error by log odds ratio for detecting publication bias and heterogeneity of preterm birth on perinatal mortality

In this study, we mostly rejected null hypotheses, and there were moderate and high levels of heterogeneity in this meta-analysis. We believe that all effect sizes in the sample of included studies might not vary only because of sampling error. As a researcher, we also anticipate the presence of unpublished studies related to perinatal mortality. It helps us think about the existence of systematic study level variability and the presence of true heterogeneity. For these reasons, selecting the random-effects model was appropriate for this meta-analysis. However, systematic review methods are subjective regarding the selection of studies to include or exclude from this review. Studies that were primarily diverse in different circumstances may lead this meta-analysis to be inaccurate. It might obscure the genuine differences in the overall mean effects of meta-analysis in the random-effect analysis. Once decisions and clinical judgments for combining individual studies are inevitably and subjectively included, there are not solutions for adjustment or amendment in statistics. It produces a wrong result interpreted as having more credibility for decision making and inappropriate summaries [51].

## Conclusion

In this review and meta-analaysis, the observed and adjusted PMR was 58.35 and 42.95 respectively per 1000 deliveries. High level of heterogeneity was evident in total studies of perinatal mortality and its determinants (I^2^ > 99 perecent). Only low birth weight and primi-parity were not approximated by statistically imputed missing studies in estimating the final effects sizes. Most determinants were presented with a positive intercept of regression and a positive correlation indicating the presence of heterogeneity and publication bias. This informs us publications existed which might be a major threat to the validity of the conclusions in this study. However, less heterogeneity was observed in subgroup analysis. Therefore, engaging in systematic review and meta-analysis would potentially improve under-represented strategies and actions by informing policy makers and program implementers for minimizing the existing socioeconomic inequalities between regions and nations. Finally, it is recommended to improve supply, demand, equity, and quality of services in countries having high perinatal mortality.

## Abbreviations

ANC: Antenatal Care
CI: Confidence Interval;
CMA: Comprehensive Meta-Analysis
DHS: Demography and Health Survey
ENAP: Early neonatal action plan
ES: Effects size
GC: Gregorian calendar
JBI: Joanna Briggs Institute
LBW: Low Birth Weight
LMICS: Low and Middle-Income Countries
PMRs: Perinatal mortality rates
POR: Pooled Odds Ratio
PRISMA: Preferred reporting items for systematic reviews and meta-analyses
SE: Standard Error
STROBE: Strengthening the Reporting of Observational Studies in Epidemiology
WHO: World Health Organization
